The article "Analysis of Clinical Efficacy of Clearing Heat and Dispelling Paralysis Soup in the Treatment of Osteoarthritis of the Knee Joint and Its Effect on Patients' Motor Function" was retracted in 2023. Reasons: signs of a paper mill; suspected computer-generated content; unreliable results or conclusions; lack of ethics approval or compliance.

# Analysis of Clinical Efficacy of Clearing Heat and Dispelling Paralysis Soup in the Treatment of Osteoarthritis of the Knee Joint and Its Effect on Patients' Motor Function

**DOI:** 10.1155/2022/5104121

**Published:** 2022-02-21

**Authors:** Lihu Xie, Mei Li

**Affiliations:** The First Affiliated Hospital, Department of Rheumatology and Immunology, Hengyang Medical College, University of South China, Hengyang Hunan 421001, China

## Abstract

**Objective:**

To investigate the effects of clearing heat and dispelling paralysis soup for osteoarthritis of the knee joint on the motor function of the knee joint and the level of inflammation of the organism in patients.

**Methods:**

One hundred and sixteen patients with knee osteoarthritis admitted from January 2020 to May 2021 were selected and randomly divided into 2 groups, 58 cases in the control group were treated with loxoprofen sodium dispersible tablets, and 58 cases in the experimental group were treated with Qinghe dispel paralysis soup on the basis of the control group and the patients' balance ability analysis, gait parameter change analysis, VAS, JOA, AIMS2-SF scale assessment, and serum index. The treatment effects of the two treatment regimens were analyzed by testing.

**Results:**

The anterior-posterior axis, left-right axis, A2-A6, A4-A8, and circumferential axis of the experimental group were lower than those of the control group after treatment (*P* < 0.05); the step length of the experimental group was higher than that of the control group after treatment (*P* < 0.05), and there were no significant differences in step speed, double-support phase, and step width (*P* > 0.05), but both groups improved significantly compared with those before treatment (*P* < 0.05); the VAS score of the experimental group was lower than that of the control group after treatment. The VAS scores of the experimental group were lower than those of the control group, and the scores of JOA and AIMS2-SF were higher than those of the control group (*P* < 0.05); the levels of TIMP-1 in the experimental group were higher than those in the control group, and the levels of TNF-*α*, TLR4, MMP-3, and IL-1 were lower than those in the control group after treatment (*P* < 0.05); there was no significant difference in the incidence of adverse reactions between the two groups during treatment (*P* > 0.05), and the efficiency of the experimental group was higher than that of the control group (*P* < 0.05).

**Conclusion:**

Combined treatment with Qinghe dispel paralysis soup can better promote the recovery of balance, improve motor ability, and reduce the development of inflammation in the organism, with high safety and effectiveness.

The article "Analysis of Clinical Efficacy of Clearing Heat and Dispelling Paralysis Soup in the Treatment of Osteoarthritis of the Knee Joint and Its Effect on Patients' Motor Function" was retracted in 2023. Reasons: signs of a paper mill; suspected computer-generated content; unreliable results or conclusions; lack of ethics approval or compliance.

## 1. Introduction

The development of osteoarthritis of the knee joint is based on degenerative pathological changes, and the main clinical manifestations of the disease are redness, swelling, and limitation of movement in the knee joint. If not treated effectively and promptly, the disease can cause joint deformity or even disability, posing a serious threat to patients' quality of life [1]. Knee osteoarthritis can be caused by overexertion, trauma, weight, walking posture, and degenerative disease, and the treatment of this disease in Western medicine is primarily anti-inflammatory and pain relief, which does not treat the disease fundamentally, and patients develop complications such as peptic ulcers and renal impairment over time [2]. Internal Chinese medicine therapy has garnered more clinical attention in recent years. Osteoarthritis of the knee joint is classified as “paralysis” in Chinese medicine and is caused by insufficient qi and blood, wind invasion, cold and dampness, and meridian stasis and should be treated with prescriptions for removing paralysis, relieving pain, and clearing dampness and heat [3].

Qinghe dispel paralysis soup is a common Chinese medicine formula that promotes qi and relieves pain, dispels wind and dampness, strengthens the spleen, and dries dampness, among other things. It has shown to be effective in the treatment of a variety of diseases. The effect of Qinghe dispelling paralysis soup on the improvement of patients' symptoms and motor functions was investigated in this study, which included 116 patients with osteoarthritis of the knee joint who were admitted to our hospital.

## 2. Materials and Methods

### 2.1. Data

One hundred and sixteen patients with knee osteoarthritis admitted to our hospital from January 2020 to May 2021 were selected and divided into two groups according to random number, 58 cases in the control group were treated with loxoprofen sodium dispersible tablets for Western medicine, and 58 cases in the experimental group were treated with clearing heat and dispelling paralysis soup on the basis of the control group. The control group was 39-72 years old, with an average age of 56.45 ± 3.53 years, 32 males and 26 females, and the duration of the disease was 1-89 months, with an average duration of 43.54 ± 1.53 months. The experimental group was 42-75 years old, mean age 57.34 ± 5.98, 33 males and 25 females, duration of illness 1-84 months, mean duration of illness 45.12 ± 4.23 months, no difference between the two groups (*P* > 0.05), and comparable data.

Inclusion criteria were as follows: (1) patients met the diagnostic criteria of osteoarthritis of the knee [4]; (2) patients met the syndromes of the Clinical Research Guidelines for New Chinese Medicines for Osteoarthrosis [5]; (3) morning stiffness of 30 min and less and frictional sounds when the joint was present; (4) X-ray showed joint space narrowing in weight-bearing position; and (5) informed and agreed to this study.

The article "Analysis of Clinical Efficacy of Clearing Heat and Dispelling Paralysis Soup in the Treatment of Osteoarthritis of the Knee Joint and Its Effect on Patients' Motor Function" was retracted in 2023. Reasons: signs of a paper mill; suspected computer-generated content; unreliable results or conclusions; lack of ethics approval or compliance.

Exclusion criteria were as follows: (1) comorbid other rheumatic diseases; (2) with severe osteoporosis; (3) with active gastrointestinal disease; (4) significant deformation of the knee joint; and (5) presence of psychiatric disorders or poor compliance. This study was approved by the ethics committee.

### 2.2. Intervention Methods

The control group received oral loxoprofen sodium dispersible tablet treatment (State Drug Quantifier: H20163219, Product No.: A14202666762, Shandong Yuxin Pharmaceutical Co., Ltd.), 60 mg/d, 3 times/d, while instructing patients to perform basic functional exercises: (1) straighten the knee joint, take the patient in the supine position, tense the quadriceps muscle, and maintain the position; (2) bend the knee and raise the hip, take the supine position, then straighten the knee joint until there is feeling of soreness and swelling, and then recover; repeat the exercise 5-10 times; (3) take the supine position, raise the legs, and perform the air pedal bicycle action, 20-30 times; (4) sit on the edge of the bed; straighten the legs, the knee joint on the bed, until there is feeling of soreness and swelling; and then bend the knee; do it continuously several times; (5) stand facing the wall, lift the heels, keep the toes on the ground, and stand; recover after soreness. All exercises were performed once a day.

On the basis of the control group, the experimental group was given Chinese herbal soup, and the formula for clearing heat and dispelling paralysis was chosen for treatment: 10 g turmeric, bitter almond, antifeng, Gentiana, earthworm, Atractylodes, and Buddha's hand; 15 g forsythia, mulberry, chicken blood vine, luo shi vine, and sea wind vine; and 5 g muxiang, one dose per day, with water decoction, concentrated to 400 ml, and divided into two doses in the morning and evening.

### 2.3. Observed Indicators

#### 2.3.1. Patient Balance Capacity Analysis

The balance ability test is conducted by dynamic balance function tester, and the main items include the left and right axis, front and back axis, peripheral axis, A2-A6 axis, and A4-A8 axis index.

#### 2.3.2. Analysis of Changes in Gait Parameters

The assessment index contains gait speed, stride length, stride width, and double-support phase, and the patient's walking ability is tested using a three-dimensional gait testing system.

#### 2.3.3. Visual Pain Analogue Rating Scale (VAS) [6]

The score was set to 0-10, with 0 indicating no pain and 10 indicating unbearable pain, and the higher the score obtained, the more obvious the patient's pain was.

The article "Analysis of Clinical Efficacy of Clearing Heat and Dispelling Paralysis Soup in the Treatment of Osteoarthritis of the Knee Joint and Its Effect on Patients' Motor Function" was retracted in 2023. Reasons: signs of a paper mill; suspected computer-generated content; unreliable results or conclusions; lack of ethics approval or compliance.

#### 2.3.4. Japanese Orthopaedic Association (JOA) [7] Score

The score mainly contains four items: daily activity ability, subjective symptoms, clinical signs, and bladder function, and the score is set from 0 to 29; the more obvious the patient's functional impairment, the lower the score.

#### 2.3.5. Arthritis Quality of Life Scale (AIMS2-SF) [8]

The scale contains 26 entries, mainly related to symptoms, somatic, emotional, work, and social, and all entries are rated on a four-point scale with scores set on a scale of 1-4, with higher quality of life patients scoring higher.

#### 2.3.6. Serum Index Tests

Five milliliters of fasting venous blood was drawn and centrifuged at 3600 rpm for 14 min to detect Toll-like receptor 4 (TLR4), tumor necrosis factor-*α* (TNF-*α*), recorded interleukin-1 (IL-1), matrix metalloproteinase-3 (MMP-3), and matrix metalloproteinase-1 (MMP-1) as well as matrix metalloproteinase inhibitor (TIMP-1), which were performed by enzyme-linked immunosorbent assay, strictly according to the instructions.

#### 2.3.7. Efficacy Analysis

The efficacy was classified according to the efficacy assessment criteria of the “Guidelines for Clinical Research on New Chinese Medicines” [9] on the disease; after treatment, the patients' joint mobility returned to normal and the pain symptoms disappeared as clinical control; the patients' joint mobility was not restricted, and the clinical symptoms disappeared as apparently small; the joint mobility was slightly restricted, and the clinical symptoms were significant. Based on the statistical findings, the effective rate was computed.

### 2.4. Statistical Methods

Data were analyzed using statistical SPSS 22.0 software, and if the data conformed to normal distribution, the count data were described by composition ratio and rate, the chi-square test was chosen for the analysis of between-group variability, and the measurement data were expressed as mean ± standard deviation, and *P* < 0.05 was taken as the difference was statistically significant, and the graphical software used for the study was GraphPad Prism 8.

## 3. Results

### 3.1. Comparison of Patients' Balance Ability

The anterior-posterior, left-right, A2-A6, A4-A8, and circumferential axes were lower in the experimental group than in the control group after treatment (*P* < 0.05) (Figure 1).

### 3.2. Comparison of Patient Gait Parameters

The step length in the experimental group was higher than that in the control group after treatment (*P* < 0.05), and there was no significant difference in step speed, double-support phase, and step width (*P* > 0.05), but both groups improved significantly compared with the pretreatment period (*P* < 0.05) (Figure 2).

The article "Analysis of Clinical Efficacy of Clearing Heat and Dispelling Paralysis Soup in the Treatment of Osteoarthritis of the Knee Joint and Its Effect on Patients' Motor Function" was retracted in 2023. Reasons: signs of a paper mill; suspected computer-generated content; unreliable results or conclusions; lack of ethics approval or compliance.

### 3.3. Comparison of Patients' VAS, JOA, and AIMS2-SF Scores

The experimental group had lower VAS scores and higher JOA and AIMS2-SF scores than the control group after treatment (*P* < 0.05) (Figure 3).

### 3.4. Comparison of TNF-*α*, TLR4, IL-1, MMP-3, and TIMP-1 Levels in Patients

The levels of TNF-*α*, TLR4, MMP-3, and IL-1 in the experimental group were lower than those in the control group, and the levels of TIMP-1 were higher than those in the control group after treatment (*P* < 0.05) (Figure 4).

### 3.5. Comparison of Patient Efficacy and Safety

There was only one case of vomiting in the experimental group during the treatment period, and the discomfort disappeared after timely antivomiting intervention, as shown in Table 1.

## 4. Discussion

Chondroprotective agents, anti-inflammatory and analgesic medicines, or intra-articular injections are often used in Western medicine to treat osteoarthritis of the knee joint, and individuals with severe lesions may be treated with artificial hip arthroplasty [10]. Data analysis revealed, however, that long-term drug treatment can cause gastrointe stinal reactions and increase the burden on the kidneys, whereas patients treated with surgery are more likely to experience postoperative rejection or postoperative joint loosening, which increases patient pain and lowers survival quality [11]. As a result, identifying safer and more effective treatment alternatives is critical for improving the long-term prognosis and quality of life of individuals with osteoarthritis of the knee [12]. In recent years, Chinese medicine has gained traction in the treatment of osteoarthritis of the knee, with reports indicating that Chinese medicine formulae have a superior safety profile and may effectively decrease treatment time and increase patient therapeutic result [13]. Patients with osteoarthritis of the knee joint were chosen for therapy with clearing heat and dispelling paralysis soup to see how effective it was.

Osteoarthritis of the knee joint is classified as “paralysis” in Chinese traditional medicine, as shown by ancient medical writings such as Su Wen-Paralysis Evidence and Ling Shu-Ying Wei Chapter, and its symptoms and causes are similar to those of osteoarthritis of the knee joint [14]. “Paralysis is a sign of Qi deficiency, and the fundamental pathophysiology is the invasion of damp and cold owing to Qi and blood shortage [15].” The condition damages the meridians of the knee joint, resulting in a long-term lack of moistening of the knee joint and surrounding tissues, and once the external wind and cold infiltrate the joint, it accumulates in the joint and produces discomfort if the joint does not flow smoothly [16]. The basic pathogenesis of osteoarthritis of the knee joint is dampness, heat, and deficiency, and the therapy should be based on formulae that can clear dampness and heat, eliminate discomfort, and alleviate pain [17]. In clear heat dispel palsy tang, Lian Qiao clears heat and reduces swelling, bitter almond opens the lung qi, the vine can promote the joints, and turtle worms can search the wind and pass through the ligaments to relieve pain, while other medicines can promote the flow of qi and relieve pain, dispel wind and dampness, and strengthen the spleen and dry dampness, respectively. Clear heat and dispel paralysis soup can promote cartilage repair by improving the function of chondrocytes, thus improving local microcirculation around the knee joint [18]. According to a study, formulae that improve the efficacy of osteoarthritis of the knee and promote the recovery of knee function in patients by activating blood circulation and detoxifying the liver and kidney can effectively improve the efficacy of osteoarthritis of the knee and promote the recovery of knee function in patients [19]. It has also been observed that treating individuals with osteoarthritis of the knee joint using herbal formulae in combination may help to reduce clinical symptoms and enhance joint function recovery [20]. The results showed that the anterior-posterior axis, left-right axis, A2-A6, A4-A8, and circumferential axis were lower in the experimental group than in the control group after treatment (*P* 0.05), and the step length was higher in the experimental group than in the control group after treatment (*P* 0.05), and there was no significant difference between the two groups in terms of stability and gait changes.

The article "Analysis of Clinical Efficacy of Clearing Heat and Dispelling Paralysis Soup in the Treatment of Osteoarthritis of the Knee Joint and Its Effect on Patients' Motor Function" was retracted in 2023. Reasons: signs of a paper mill; suspected computer-generated content; unreliable results or conclusions; lack of ethics approval or compliance.

Pain is the main symptomatic manifestation of osteoarthritis of the knee, and effective control of joint pain in patients is crucial to improve their survival quality. It has been pointed out in a study that herbal treatment can better control joint pain [21–23]. In this study, the VAS, JOA, and AIMS2-SF scores of patients were analyzed, and the results showed that the VAS scores of the experimental group were lower than those of the control group after treatment, and the JOA and AIMS2-SF scores were higher than those of the control group (*P* < 0.05), suggesting that the combined treatment with clearing heat and dispelling paralysis soup could better control the joint pain of patients and improve their survival quality. Inflammation development is the key to the occurrence and development of osteoarthritis disease in the knee joint [24–26]. TLR4 mainly mediates natural immune and inflammatory responses and is a pattern recognition receptor, and it has been pointed out in a study that synovial fluid in bone and joint tissues produces plasma proteins through the TLR4 pathway, which in turn leads to the development of synovitis. TNF-*α* accelerates proteoglycan degradation and inhibits cartilage collagen production. IL-1 responds to the inflammatory response of the body, and MMP-3 accumulates proteoglycans, and when the levels of both substances increase, it promotes articular cartilage damage and exacerbates the clinical symptoms of patients. It promotes inhibitory effect and promotes osteoarticular repair. In this study, the levels of inflammatory indexes in the two groups were analyzed, and the results showed that the levels of TNF-*α*, TLR4, MMP-3, and IL-1 in the experimental group were lower than those in the control group after treatment, and the levels of TIMP-1 were higher than those in the control group (*P* < 0.05), suggesting that the combined treatment with Qinghe dispel paralysis soup can better control the inflammation of the patient's organism. The complications and efficiency of the two groups of patients were analyzed to further analyze the effectiveness and safety of this experimental treatment plan, and the results showed that the experimental group's efficiency was significantly higher, and the patients had no significant complications.

To summarize, combining traditional Western medicine therapy with Qinghe dispel paralysis soup may help promote balance recovery, increase motor capacity, and limit the development of inflammation in the body while also being very safe and effective.

## Figures and Tables

**Figure 1:** Comparison of patients' balance ability.

**Figure 2:** Comparison of patient gait parameters.

**Figure 3:** Comparison of patients' VAS, JOA, and AIMS2-SF scores.

**Figure 4:** Comparison of TNF-*α*, TLR4, IL-1, MMP-3, and TIMP-1 levels in patients.

**Table 1:** Comparison of patient efficacy and safety $\left(\bar{x}\pm s\right)$.

Group	Number of cases	Clinical control	Show effect	Effective	Invalid	Efficient
Experimental group	58	12 (20.69)	18 (31.03)	25 (43.10)	3 (5.17)	55 (94.83)
Control group	58	7 (12.07)	12 (20.69)	23 (39.66)	16 (27.59)	42 (72.41)
*X* ^2^	/	5.632				
*P*	/	<0.05				

## Data Availability

The data used to support the findings of this study are included within the article.
